The article "AKAP12 and RNF11 as Diagnostic Markers of Fibromyalgia and Their Correlation with Immune Infiltration" was published in 2022. Journal: Oxid Med Cell Longev.

# AKAP12 and RNF11 as Diagnostic Markers of Fibromyalgia and Their Correlation with Immune Infiltration

**DOI:** 10.1155/2022/9033342

**Published:** 2022-10-04

**Authors:** Xiaowen Lin, Kangda Zhang, Tao Meng

**Affiliations:** ^1^Department of Pain Management, Shandong Provincial Hospital Affiliated to Shandong First Medical University, Jinan, China; ^2^Department of Anesthesiology, Qilu Hospital of Shandong University, Jinan, China

## Abstract

Fibromyalgia (FM) is a chronic nonarticular rheumatic disease mainly characterized by diffuse disseminated skeletal muscle pain, with varied symptoms including anxiety, sleep disturbance, and fatigue. Due to its unknown etiology and pathogenesis, FM is easily ignored in clinical practice, resulting in unclear diagnosis and difficult treatment. This study is aimed at investigating whether AKAP12 and RNF11 can be used as biomarkers for the diagnosis of FM and at determining their correlation with immune infiltration. The FM dataset in Gene Expression Omnibus (GEO) database was downloaded and was randomly divided into the training and test sets. Differentially expressed genes (DEGs) were screened, and functional correlation analysis was performed. Diagnostic markers of FM were screened and validated by random forest (RF). The least absolute shrinkage and selection operator (LASSO) logistic regression algorithm was then used to evaluate immune cell infiltration in the FM patients' peripheral blood. Finally, Spearman's rank correlation analysis was used to identify correlation between the diagnostic indexes and immune cell infiltration. A total of 69 DEGs were selected. Results indicated that AKAP12 and RNF11 can be used as diagnostic markers of FM, and CD8 + T cells might contribute in the pathogenesis of FM. In addition, AKAP12 was positively correlated with CD8 + T cells, while RNF11 was negatively correlated with CD8 + T cells. In conclusion, AKAP12 and RNF11 can be used as diagnostic indicators of FM, and CD8 + T cells may be involved in the occurrence and development of FM.

## 1. Introduction

Fibromyalgia (FM) is a chronic, painful, nonarticular rheumatic disease characterized by diffuse pain and often accompanied by multiple symptoms, including fatigue, sleep disturbances, emotional abnormalities, and cognitive dysfunction [1]. So far A kinase anchoring protein-12 (AKAP12) and RNF11 have not shown any abnormal expression in any osteoarthritis and rheumatoid arthritis. FM is considered the third most common musculoskeletal disorder, and its incidence increases with age [2]. Due to improved diagnosis techniques, the current FM prevalence is about 2%-8% [3]. A great controversy still exists regarding FM assessment and diagnosis. Initially, the diagnosis of FM proposed by the American College of Rheumatology (ACR) in 1990 mainly consisted of counting 18 tenderness points at the same anatomical site on the left and right sides of the body [4]. Although widespread chronic pain lasting more than 3 months is the main symptom of FM, there are still about 70%-80% of patients with specific manifestations such as sleep disturbance and lethargy, which cannot be ignored [5].

Later, in 2010, the ACR updated its diagnostic criteria, which assessed the presence and severity of fatigue, cognitive difficulties, sleep deprivation, degree of other somatic symptoms, and considered the painful body parts [6]. The ACR 2010 criteria, which rely on Symptom Severity Scale (SSS) and the Widespread Pain Index (WPI), are more sensitive than the ACR 1990 criteria and are presently widely used in clinical practice [7]. Routine clinical laboratory diagnoses of FM do not reveal objective abnormalities, and diagnosis is usually done based on complex clinical manifestations after excluding other diseases. Due to the delayed diagnosis, progression of FM in most patients leads to poor prognosis and ineffective treatment options. Consequently, exploring biomarkers might help in early diagnosis and improve prognosis.

The underlying mechanisms of FM are complex and result from the interaction of mental stress, neuroendocrine abnormalities, immune dysfunction, and behavioral and psychological factors [8, 9]. Recent studies have shown that immune cell infiltration is essential in FM occurrence and development. Blood sample immunophenotypic analysis from patients revealed the role of Mu opioid receptors on B lymphocytes as specific biomarkers for FM [10]. From the immune system perspective, it is important to evaluate the differences in immune cell components infiltrated in peripheral blood of FM patients compared to healthy people to elucidate the molecular mechanism and develop possible immunotherapeutic targets. With the widespread use of microarray and high-throughput sequencing, bioinformatics analysis can identify novel genes and biomarkers associated with various disease development, including systemic lupus erythematosus, osteoarthritis, and rheumatoid arthritis [11–13]. CIBERSORT is an analytical tool that uses gene expression profiles to assess the expression and composition of immune cells [14].

The present investigation is aimed at investigating whether AKAP12 and RNF11 can be used as biomarkers for the diagnosis of FM and at determining their correlation with immune infiltration. A microarray dataset of FM was downloaded from Gene Expression Omnibus (GEO) database to identify Differentially Expressed Genes (DEGs). After DEG screening, the functional correlation was analyzed by Gene Ontology (GO) and Kyoto Encyclopedia of Genes and Genomes (KEGG), and machine learning algorithms were used to further screen and determine diagnostic markers of FM. Subsequently, CIBERSORT was used to analyze the differences in immune cell subsets' infiltration between FM patients and healthy subjects. Finally, we investigated the relationship between diagnostic markers and infiltrating immune cells.

## 2. Materials and Methods

### 2.1. Data Download and Preprocessing

The GEO database (http://www.ncbi.nlm.nih.gov/geo) is an open-source platform created by the National Biotechnology Information Center of the United States (NCBI) to retrieve gene expression data. The GSE67311 dataset consisted of 142 whole blood samples from 67 patients with fibromyalgia syndrome and 75 healthy controls, and the results were published in 2016 by Jones et al. [15]. All subjects were genotyped using the GPL11532 Affymetrix Human Gene 1.1 ST Array. After downloading the raw gene expression data, it was standardized using a robust multiarray averaging (RMA) algorithm, and 142 samples were randomly divided into the training and test sets. The training set consisted of 95 samples for screening differential and characteristic genes. The test set had 47 samples for validating the analysis results. All statistical analyses were performed using the R software (version 3.6.3).

### 2.2. DEG Identification

After data were standardized, the “limma” package was used to identify DEGs between FM patients and healthy controls [16]. DEGs with *P* < 0.05 and |log_2_*FC*| > 0.2 were considered statistically significant [17]. The volcano map of DEGs was drawn using the “ggplot2” package.

### 2.3. Functional Enrichment Analysis

The “clusterProfiler” package was used for GO and KEGG enrichment analyses to explore the potential biological functions of DEGs in patients and healthy controls [18]. GO terms include biological process (BP), cellular component (CC), and molecular function (MF). The significance threshold of GO analysis was set as an adjusted *P* value < 0.05, and KEGG analysis was set as *P* value < 0.05. The above analysis results are presented as a bar chart and bubble chart by the “ggplot2” package.

### 2.4. Screening and Verification of Diagnostic Markers

As a technical means to achieve artificial intelligence (AI), machine learning can automatically analyze existing data to obtain rules or models and use the guidelines to predict unknown data [19]. Here, we applied a computational method combining random forest (RF) and least absolute shrinkage and selection operator (LASSO) logistic regression algorithms to screen genetic biomarkers of FM and construct diagnostic models. We specifically used “glmnet” package for LASSO analysis and the “randomForest” package for random forest algorithm analysis [20, 21]. We obtained diagnostic marker genes that overlapped with LASSO and the random forest algorithm. The sensitivity and specificity of the diagnostic prediction model were analyzed by the receiver operating characteristic (ROC) curve and quantified by the area under ROC curve (AUC). Next, we verified the test set and reserved the gene with AUC greater than 0.6 as the final diagnostic marker gene.

### 2.5. Evaluation of Immune Cell Subtype Distribution

CIBERSORT (http://CIBERSORT.stanford.edu/) was used to evaluate the proportion of 22 subtypes of immune cells in the human body, while the LM22 signature matrix was used to define 22 infiltrating immune cells components. After obtaining the immune cell infiltration matrix, the Wilcoxon test was used to screen different immune cell infiltration between FM patients and normal controls. *P* < 0.05 was considered statistically significant, and the results were presented in a boxplot. The correlations of 22 infiltrating immune cells were analyzed using the “corrplot” package [22].

### 2.6. Correlation Analysis between Diagnostic Biomarkers and Immune Cells

Spearman correlation test was used to analyze the correlation between the immune score of characteristic immune cells and the expression level of diagnostic marker genes. The results were visualized by the “ggplot2” package.

## 3. Results

### 3.1. Identification of DEGs

DEGs were shown in the volcano map (Figure 1). Compared with healthy controls, FM patients had 26 upregulated DEGs and 43 downregulated DEGs.

### 3.2. Functional Enrichment Analysis

The high-throughput data analysis allows us to obtain several candidate genes. To better understand the function of these genes, we used enrichment analysis, which reflects them as a whole. GO analysis results showed that DEGs were mainly related to defense response to the virus, regulation of viral genome replication, type I interferon (IFN) signaling pathway, and cellular response to type I IFN (Figures 2(a) and 2(b)). Furthermore, the KEGG enrichment analysis suggested that the map05167 pathways of herpes simplex virus 1 (HSV-1) infection might be the biological pathways altered in FM patients compared with healthy controls (Figures 2(c) and 2(d)).

### 3.3. Screening and Verification of Diagnostic Markers

We first used a random forest algorithm to identify 4 genes from DEGs as diagnostic markers of FM (Figure 3(a)) and made a ROC curve (Figure 3(b)). Nineteen DEGs were then screened by the LASSO regression algorithm (Figures 3(c) and 3(d)). The marker genes obtained by the two algorithms were overlapped to obtain 4 diagnostic characteristic genes, namely, AKAP12, CCR9, IL3RA, and RNF11. In order to further test the diagnostic efficacy of the above genes, test sets were used to verify them. ROC analysis was performed by the R software to predict the diagnostic effectiveness of biomarkers, and only genes with AUC > 0.6 were retained as the final marker genes. The results showed that AKAP12 (AUC = 0.628) and RNF11 (AUC = 0.663) had high diagnostic values. We combined genes and observed that AUC was also greater than 0.6 when CCR9 was combined with RNF11 (AUC = 0.643) and AKAP12 was combined with IL3RA (AUC = 0.617) (Figure 4).

### 3.4. Immune Cell Infiltration in FM and Its Relationship with Diagnostic Markers

The correlation of 22 groups of immune cells in the blood of FM patients was first evaluated (Figure 5(a)). According to the results, M1 macrophages, activated mast cells, resting mast cells, plasma cells, regulatory T cells, M2 macrophages, activated dendritic cells, memory B cells, Th cells, activated NK cells, and resting dendritic cells had a significant positive correlation. Resting CD4 memory T cells and neutrophils had a significant negative correlation. The Wilcoxon test was then used to evaluate significant differences in immune cell infiltration in peripheral blood between FM patients and the control group.  Figure 5(b) shows the different immune cell occupation in peripheral blood of FM patients and healthy controls. CD8+ T cells were significantly reduced in FM patients compared with the control group, confirming the importance of reducing this cell type in the FM immune microenvironment. Furthermore, the correlation among four effective biomarkers (AKAP12, CCR9, IL3RA, and RNF11) and one significantly differential immune cell (CD8+ T cells) is presented in Figure 6(a). Correlation analysis showed that AKAP12 was positively correlated with CD8+ T cells (*R* = 0.33, *P* = 0.0012), while RNF11 was negatively correlated with CD8+ T cells (*R* = −0.34, *P* = 0.00066) (Figures 6(b) and 6(c)).

## 4. Discussion

Fibromyalgia has been broadly described as a multifaceted disease, including autoimmune, infectious, and somatic disorders [23]. Due to the various symptoms and lack of early diagnostic indicators, FM patients are often only diagnosed after excluding other diseases, leading to late treatment. According to evidence, inflammation plays a role in fibromyalgia pathogenesis [24–26]. Research on suitable specific diagnostic markers and the infiltrating immune cell landscape identification helps consolidate the prognosis of FM patients. In this study, bioinformatics was used to screen molecular markers of FM. CIBERSORT analysis facilitated the analysis of immune cell infiltration patterns in the disease. We focused on identifying the diagnostic markers and exploring the role of immune cell infiltration in FM.

The FM gene expression dataset from the GEO database was downloaded and randomly divided into the training and test sets to select the optimal model. Under the differential expression threshold, 69 DEGs were identified. GO and KEGG analyses were performed on DEGs to decipher the underlying biological mechanisms contributing to FM progression. The results of GO analysis showed that DEGs were mainly involved in virus defense response and IFN signaling pathway. KEGG analysis showed that enriched pathways mainly involved the HSV-1 infection pathway. Sarzi-Puttini et al. evaluated the efficacy of an antiherpetic drug in combination with a COX-2 inhibitor (famciclovir + celecoxib, IMC-1) in FM patients in a 16-week double-blind, placebo-controlled trial conducted at 12 centers [2]. Compared with placebo, the IMC-1-treated patients had a significantly reduced FM-related pain, improved Patient's Global Impression of Change (PGIC) response rates, better self-reported function as measured by the Revised Fibromyalgia Impact Questionnaire (FIQ-R), and reduced fatigue as measured by the NIH Patient-Reported Outcomes Measurement Information System (PROMIS). In contrast, neither drug alone seemed to relieve symptoms of FM. Their results support the hypothesis that HSV infection may cause FM and are consistent with our analysis.

In order to improve the accuracy of the results, two independent machine learning algorithms (RF and LASSO logistic regression) were used to screen various variables and establish the optimal classification model. Finally, four DEGs (AKAP12, CCR9, IL3RA, and RNF11) were identified and verified by the test set as diagnostic markers of FM. The validation of AKAP12 and RNF11 seems to be reliable, indicating that the strategy for modeling is feasible. According to previous reports, RING finger protein 11 (RNF11), a 154 amino acid protein belonging to the E3 ubiquitin ligase family, is strongly associated with human breast cancer and hepatocellular carcinoma [27–29]. As a posttranslational modification of proteins, ubiquitination controls almost all cellular processes, explaining the diversity of ubiquitination in different cellular pathways. Ubiquitination requires sequence action of E1 ubiquitin-activating enzyme, E2 ubiquitin-conjugating enzyme, and E3 ubiquitin-protein ligase to bind the ubiquitin chain to the target protein, resulting in protein degradation or protein stabilization [30]. However, the mechanism used by RNF11 to regulate protein ubiquitination remains unclear because the RNF11 promotes ubiquitination in some cases but inhibits substrate ubiquitination in other instances [31]. Hsu et al. conducted a metabolomic and proteomic analysis of serum samples from patients with FM, and the results showed that FM patients had metabolic disorders and produced numerous NF-*κ*B-dependent cytokines [32]. RNF11 has been reported as a negative regulator of NF-*κ*B and Jun N-terminal kinase (JNK) signaling pathways [33]. Another study reported that RNF11 negatively regulates the inflammatory signaling pathway of microglia, which may be a potential target for regulating neuroinflammatory responses [34]. RNF11 upregulation may protect neurons from nonregulated inflammation [35]. In our study, the increased expression of RNF11 in peripheral blood cells of FM patients might have upregulated inflammation.

AKAP12, an anchor gene that mediates the subcellular compartmentation of protein kinase A (PKA) and protein kinase C (PKC), was initially identified as a molecule associated with poor prognosis in myasthenia gravis [36]. Subsequently, AKAP12 was found to inhibit malignant tumor metastasis and progression, regulate the formation of blood-brain and blood-retinal barriers, and resensitize *β*2-adrenergic pain receptors [37]. Since sleep dysfunction has been shown to reduce descending spinal inhibition of pain signals [38], a significant difference in the frequency of Gly16Arg polymorphism in the *β*2-adrenergic receptor gene was observed in FM patients with varying degrees of sleep disorders compared to the controls [39]. AKAP12 expression may be negatively correlated with estrogen levels, and in granulosa cells with estrogen receptor- (ER-) *β* deletion, AKAP12 is upregulated after FSH treatment [40]. In our study, AKAP12 was downregulated in FM patients, which seems to confirm that FM prevalence is higher in females than males. However, big cohort studies are still needed to confirm the diagnostic value of AKAP12 and RNF11 in peripheral blood.

Previous works of literature are inconclusive on the role of immune cell infiltration in FM development and maintenance. Consequently, this investigation used CIBERSORT online tool to evaluate immune infiltration of FM comprehensively. CD8 + T cells were significantly downregulated in FM patients compared to the control group. In addition, the correlation analysis showed that CD8 + T cells were positively correlated with RNF11 and AKAP12. Nishikai et al. reported antibodies against 68/48 kDA protein in some patients with chronic fatigue syndrome and primary FM, which might confirm FM as an immune-mediated disease [41]. The coexistence of endometriosis and FM is associated with a high burden of autoimmune diseases, depression, and anxiety [42].

Further, B or T cell-mediated cross-reactive responses may occur in chronic pain and systemic inflammation, but recent research on the association between FM and adaptive immunity seems to focus on CD4 + T cells [43]. However, serum CD8 + T cell levels were lower in chronic pain patients than in healthy subjects [44]. A study investigating the effects of pain and stress on lymphocyte count and lymphocyte subsets showed that the number of cytotoxic CD8+ lymphocytes was significantly reduced in patients with chronic pain, while the CD4/CD8 ratio was not significantly changed. Posttraumatic stress score was negatively correlated with the number of CD8 + T cells in FM patients [45]. Therefore, the immune system is no longer a bystander in the occurrence and maintenance of FM. The pathophysiological mechanism of FM and the formation of general inflammation may also involve adaptive immune cells, especially T cells, which need further study.

We innovatively adopted machine learning methods based on current sample GitHub to screen and verify the diagnostic markers of FM, which need to further improve the predictive algorithms. CIBERSORT was used to analyze the infiltration of immune cells in the peripheral blood of FM. However, we acknowledge that this study has some limitations. Firstly, our analysis is secondary mining of previously published data sets, and different conclusions may be drawn due to the differences in analytical ideas and perspectives. Secondly, this study lacks relevant clinical information and self-sequencing test, which will be the direction of our future clinical research on FM. Thirdly, the CIBERSORT algorithm is only based on limited transcriptome data, and the distribution of some low abundance expressed immune cell subsets in FM has not been fully revealed. As a result, our research results are not only consistent with some previous studies but also contradictory to some of them. The limitations of this study require further laboratory validation.

## 5. Conclusion

In summary, bioinformatics analysis confirmed that peripheral blood RNF11 and AKAP12 might be used as diagnostic markers of FM. In addition, CD8 + T lymphocytes might play a role in the occurrence and development of FM and are significantly correlated with RNF11 and AKAP12. Therefore, this study may provide a new perspective on the diagnosis of FM, especially from the aspects of immune cells and immune regulation.

## Figures and Tables

**Figure 1:** Volcano map of DEGs. Red represents high expression, blue represents low expression, and gray represents no difference.

**Figure 2:** GO and KEGG functional enrichment analyses of DEGs. (a) Histogram of GO enrichment analysis. (b) Bubble plot for GO enrichment analysis. (c) Histogram of KEGG enrichment analysis. (d) Bubble plot for KEGG enrichment analysis.

**Figure 3:** Diagnostic gene screening process. (a) The cross-validation curve of the relationship between model error and the number of genes used for fitting. (b) The ROC curve of signature genes is screened by a random forest algorithm. (c) LASSO coefficient profiles of the nineteen potential genes. (d) The partial likelihood deviation curve of the minimum number of signature genes.

**Figure 4:** ROC curve to verify the diagnostic efficacy of candidate genes.

**Figure 5:** Immune cell infiltration. (a) The correlation of 22 immune cells in peripheral blood of patients with FM was evaluated. Red is positive, and blue is negative. (b) The box diagram shows the proportion of 22 groups of immune cells in the peripheral blood of FM patients and healthy persons.

**Figure 6:** Correlation between diagnostic markers and differential immune cells in FM. (a) Correlation among 4 diagnostic biomarkers and CD8+ T cells. (b) Correlation between CD8+ T cells and AKAP12. (c) Correlation between CD8+ T cells and RNF11. *P* < 0.01.

## Data Availability

All data, models, and code generated or used during the study appear in the submitted article.
